# Preparation of Inactivated Human Skin Using High Hydrostatic Pressurization for Full-Thickness Skin Reconstruction

**DOI:** 10.1371/journal.pone.0133979

**Published:** 2015-07-30

**Authors:** Pham Hieu Liem, Naoki Morimoto, Atsushi Mahara, Chizuru Jinno, Koji Shima, Shuichi Ogino, Michiharu Sakamoto, Natsuko Kakudo, Masukazu Inoie, Kenji Kusumoto, Toshia Fujisato, Shigehiko Suzuki, Tetsuji Yamaoka

**Affiliations:** 1 Department of Plastic and Reconstructive Surgery, Graduate School of Medicine, Kyoto University, Kyoto, Japan; 2 Department of Plastic and Reconstructive Surgery, Kansai Medical University, Hirakata, Japan; 3 Department of Biomedical Engineering, National Cerebral and Cardiovascular Center Research Institute, Suita, Japan; 4 Department of Biomedical Engineering, Osaka Institute of Technology, Osaka, Japan; 5 Japan Tissue Engineering Co., Ltd., Gamagori, Japan; 6 Department of Plastic and Aesthetic Surgery, Pham Ngoc Thach University of Medicine, Ho Chi Minh City, Vietnam; Institute for Frontier Medical Sciences, Kyoto University, JAPAN

## Abstract

We have reported that high-hydrostatic-pressure (HHP) technology is safe and useful for producing various kinds of decellularized tissue. However, the preparation of decellularized or inactivated skin using HHP has not been reported. The objective of this study was thus to prepare inactivated skin from human skin using HHP, and to explore the appropriate conditions of pressurization to inactivate skin that can be used for skin reconstruction. Human skin samples of 8 mm in diameter were packed in bags filled with normal saline solution (NSS) or distilled water (DW), and then pressurized at 0, 100, 150, 200 and 1000 MPa for 10 minutes. The viability of skin after HHP was evaluated using WST-8 assay. Outgrowth cells from pressurized skin and the viability of pressurized skin after cultivation for 14 days were also evaluated. The pressurized skin was subjected to histological evaluation using hematoxylin and eosin staining, scanning electron microscopy (SEM), immunohistochemical staining of type IV collagen for the basement membrane of epidermis and capillaries, and immunohistochemical staining of von Willebrand factor (vWF) for capillaries. Then, human cultured epidermis (CE) was applied on the pressurized skin and implanted into the subcutis of nude mice; specimens were subsequently obtained 14 days after implantation. Skin samples pressurized at more than 200 MPa were inactivated in both NSS and DW. The basement membrane and capillaries remained intact in all groups according to histological and immunohistological evaluations, and collagen fibers showed no apparent damage by SEM. CE took on skin pressurized at 150 and 200 MPa after implantation, whereas it did not take on skin pressurized at 1000 MPa. These results indicate that human skin could be inactivated after pressurization at more than 200 MPa, but skin pressurized at 1000 MPa had some damage to the dermis that prevented the taking of CE. Therefore, pressurization at 200 MPa is optimal for preparing inactivated skin that can be used for skin reconstruction.

## Introduction

Skin consisting of the epidermis and the dermis is the largest organ in the body and protects the body against heat, desiccation and infection. It consists of the epidermis and the dermis. As for skin regeneration, the epidermis can be regenerated using cultured epidermis (CE) by Green’s method [1,2]. However, regeneration of the dermis with sufficient strength and elasticity has yet to be realized. Dermal substitutes composed of collagen matrix have been used clinically, however, the strength and elasticity of regenerated dermis-like tissue are still controversial [3]. Decellularized dermis could be an ideal dermal substitute because its structure and mechanical properties are those of the native dermis itself. Various decellularization methods have been reported and chemical methods such as the use of hypertonic solution, detergent treatment or enzymatic digestion have been widely used [4–6]. These methods require several days for the inactivation process and several weeks for washing out the debris of cells. Sodium dodecyl sulfate (SDS) is reported to be effective and clinical cases using this method have been reported [7,8]. However, SDS was reported to have cytotoxicity and our previous study showed that human cultured epidermis did not take on dermis decellularized using SDS [9].

We have reported that high-hydrostatic-pressure (HHP) technology is a safe decellularization method without detergents and that this method successfully decellularized various kinds of decellularized tissue, such as a heart valve [10], blood vessel [11], cornea [12] and bone [13]. As for the effect of hydrostatic pressure on cell viability, we reported that pressure of 200 MPa for 10 min was sufficient to induce cell killing through the inactivation of mitochondrial activity [14] and inactivated porcine skin completely without damaging the extracellular matrix [15]. In this study, we pressurized human skin and explored the appropriate pressure for inactivating human skin that can be used for skin reconstruction. Excessive pressure has the potential to disrupt the structure of the extracellular matrix through protein denaturation; therefore, we also explored the adhesion of cultured epidermis to pressurized skin in order to evaluate the possibility of using pressurized skin for skin reconstruction.

## Materials and Methods

### 1. Ethics statement

Our protocol was approved by the ethics committee of Kyoto University Graduate School Faculty of Medicine (the approval number: E1050). Skin specimens were obtained from patient volunteers with written informed consent. Our experimental protocol was approved by the Animal Research Committee, Kyoto University Graduate School of Medicine. Animal experiments were performed at Kyoto University. The number of animals used in this study was kept to a minimum and all possible efforts were made to reduce their suffering in compliance with the protocols established by the Animal Research Committee.

### 2. Preparation of human skin

Skin specimens were obtained from four female patient volunteers (mean age: 46.75 years old, range: 46–52 years old) who underwent reconstructive breast surgery using deep inferior epigastric perforator flaps at Kyoto University Hospital. Skin was preserved in normal saline solution (NSS; Otsuka Pharmaceutical Ltd., Tokyo, Japan) at 4°C, subcutaneous tissue was removed with scissors and full-thickness skin of 8 mm in diameter was prepared using 8 mm biopsy punches (Kai Industries Co., Ltd., Gifu, Japan).

### 3. Pressurization of skin

Our HHP procedure is summarized in Table 1. After packing specimens of each group in a plastic bag filled with NSS or DW (Otsuka Pharmaceutical Ltd., Tokyo, Japan), the bag was immersed in transmission fluid in the chamber of a cold isostatic pressurization machine (Dr. CHEF, Kobe Steel, Ltd., Kobe, Japan). NSS or DW was used as a solution during pressurization and specimens were pressurized at 0, 100, 150, 200 and 1000 MPa using the machine. Skin specimens were divided into 10 groups (n = 16 in each group) according to the solution and pressure (NSS-0, NSS-100, NSS-150, NSS-200, NSS-1000, DW-0, DW-100, DW-150, DW-200 and DW-1000). The pressure was increased from 0 (without pressurization) to 100, 150, 200 and 1000 MPa at a rate of 65.3 MPa/min at 30°C and kept there for 10 min. Then, the pressure was decreased at the same rate [12–15].

**Table 1:** Our HHP procedure.

1. Pack specimens in a plastic bag filled with NSS or DW
2. Immerse the bag in transmission fluid in the chamber of a cold isostatic pressurization machine (Dr. CHEF)
3. Increase the pressure from 0 to 100, 150, 200 and 1000 MPa at a rate of 65.3 MPa/min at 30°C
4. Maintain the target pressure for 10 min
5. Decrease the pressure at a rate of 65.3 MPa/min

### 4. Evaluation of the viability of pressurized skin

The viability of pressurized skin was evaluated by WST-8 (4-[3-(2-methoxy-4-nitro-phenyl)-2-[4-nitrophenyl]-2H-5-tetrazolio]-1,3-benzene disulfonate sodium salt) assay (Cell Count Reagent SF, Nacalai Tesque, Co., Ltd., Kyoto, Japan). This assay is a modified version of the MTT (3-[4,5-dimethylthiazol-2-yl]-2,5-diphenyltetrazolium bromide) assay and a colorimetric assay [16]. Immediately after pressurization, 2 specimens of 3 mm in diameter (n = 6 in each group) were obtained from each sample of 8 mm in diameter (n = 3 in each group) using 3 mm biopsy punches (Kai Industries Co., Ltd., Gifu, Japan). Each sample was placed into a well of a 96-well plate (Nunc Co., Roskilde, Denmark) and 100 μl of Dulbecco’s modified Eagle’s medium (DMEM, Life Technologies Co., Tokyo, Japan) was added to each well and incubated for 15 minutes at 37°C. Then, 10 μl of the test reagent was added and incubated for 1 hour at 37°C. Next, specimens were removed and the absorbance of the medium was read using a microplate reader (model 680; Bio-Rad Laboratories, Inc., Hercules, CA) at a test wavelength of 450 nm and a reference wavelength of 650 nm. The mean absorbance of the DMEM (n = 6) was used as an arbitrary zero point.

### 5. Outgrowth culture of the pressurized skin and its viability after cultivation

Two specimens of 3 mm in diameter (n = 6 in each group) were obtained from each pressurized skin sample, as mentioned above. Each sample was placed in a well of a collagen type I-coated 24-well plate (AGC Techno Glass Co., Ltd., Japan) and a glass slide of approximately 1 x 1 cm was placed on each specimen to prevent it from floating. A total of 1 ml of High-Glucose DMEM (Life Technologies Co., Japan, Tokyo, Japan) with 10% fetal bovine serum (FBS, Life Technologies Co., Japan, Tokyo, Japan) and with 100 units/mL penicillin, 100 μg/mL streptomycin and 250 ng/mL amphotericin B (Life Technologies Co., Japan, Tokyo, Japan) was added to each well and incubated at 37°C, 95% humidity and 5% carbon dioxide. The medium was changed every three days. After 2 weeks, specimens were removed from the wells and migrated fibroblasts were observed using an optical microscope (TS1F-APH, NIKON, Co., Tokyo, Japan) at 200x magnification. Then, the levels of viability of skin were evaluated using WST-8 assay. Each specimen was placed into a well of a 96-well plate and 100 μl of DMEM was added and incubated for 15 minutes at 37°C. A total of 10 μl of the test reagent was added and incubated for 1 hour at 37°C. Next, the absorbance was read at a test wavelength of 450 nm and a reference wavelength of 650 nm. DMEM alone was used as a control.

### 6. Histological and immunohistochemical examination of the basement membrane and capillaries of pressurized skin

The pressurized skin was fixed with 10% neutral-buffered formalin solution and embedded in paraffin blocks; the central area of each sample was then sectioned at 5 μm thickness following hematoxylin and eosin (HE) staining. Microphotographs were taken using a fluorescent microscope (Biorevo BZ-9000; Keyence, Co., Osaka, Japan). Other 5-μm-thick sections were used for immunohistochemical staining of type IV collagen for the basement membrane of epidermis and capillaries, and immunohistochemical staining of von Willebrand factor (vWF) for capillaries. After deparaffinization and rehydration, antigen retrieval processing was performed using the heat-induced target retrieval method. The sections were immersed in a pre-heated staining dish containing a modified citrate buffer (pH 6.1; Dako Japan Co., Tokyo, Japan) and incubated for 30 minutes at 90°C. After being cooled to room temperature, the sections were rinsed twice in PBS and immersed in 130 ml of methanol (CH_3_OH; Wako Pure Chemical Industries Ltd., Osaka, Japan) mixed with 4 ml of hydrogen peroxide (H_2_O_2_; Wako Pure Chemical Industries Ltd., Osaka, Japan) for 10 minutes to block endogenous peroxidase activity. To block non-specific protein binding, protein blocking agent (PBA; Thermo Ltd., California, U.S.A.) was applied for 10 minutes. Next, the sections were incubated with rabbit polyclonal anti-type IV collagen antibody (dilution 1:500; Abcam Co., Ltd., Boston, U.S.A.) or rabbit polyclonal anti-human vWF antibody (dilution 1:300; Dako Japan Co., Ltd., Tokyo, Japan) as primary antibodies at room temperature for 30 minutes. Then, the peroxidase-labeled secondary antibody, MAX PO (multi) (Nichirei Biosciences Co., Ltd., Tokyo, Japan), was applied and incubated for 30 minutes. The sections were rinsed with PBS and exposed to DAB (3–3’-diaminobenzidine tetrahydrochloride; Dako Japan Co., Ltd., Japan) and counterstained with hematoxylin.

### 7. Scanning electron microscopy (SEM)

Specimens were fixed in glutaraldehyde (2% in 0.1 M cacodylate buffer, pH 7.4), dehydrated in a graded series of ethanol, and dried in a *t*-butanol dryer. Each section was coated with platinum in a coater (JFC-1600, JEOL, Tokyo, Japan) and observed by SEM (JSM-6390LV, JEOL, Tokyo, Japan).

### 8. Implantation of pressurized skin into nude mice

Seven-week-old male BALB/c nude mice (n = 20; Shimizu Laboratory Supply, Kyoto, Japan) were used. The mice were anesthetized via the intraperitoneal injection of sodium pentobarbital (40 mg/kg; Dainippon Sumitomo Pharmaceutical Co. Ltd., Osaka, Japan). Pressurized skin samples of 8 mm in diameter were implanted into the subcutis of both sides of the mice (n = 4 in each group, 2 pieces per mouse). Mice were sacrificed by carbon dioxide inhalation and specimens were taken 14 days after implantation. Specimens were frozen and mounted using O.C.T. compound (Sakura Fine Technical Co., Ltd., Tokyo, Japan), and 5-μm-thick frozen sections were prepared from the central area of each specimen, fixed with 10% formaldehyde and subjected to HE staining.

### 9. Implantation of pressurized skin with cultured epidermis (CE) into nude mice

Human CE using keratinocytes cultured from human neonatal foreskin was prepared by Japan Tissue Engineering (J-TEC Co., Ltd., Gamagori, Japan). In preparation, J-TEC used the same Green’s method to prepare autologous CE product in Japan. Keratinocytes were labeled with PKH26 (Sigma Chemical, St. Louis, MO), a red fluorescent dye that emits at 567 nm, according to the manufacturer’s protocol, at the last passage. In the previous experiments, epidermis was not observed after pressurization at 150, 200 and 1000 MPa in NSS and 100, 150, 200 and 1000 MPa in DW. CE was cut to a square 10mm×10mm in size by scissors. Each CE was raised and putted on the pressurized skin (n = 4 in each group) using forceps. Then, the pressurized skin with CE was implanted into the subcutis of nude mice as in the previous experiment. Mice were sacrificed 14 days after implantation and 5-μm-thick frozen sections were prepared from the central area of each specimen. After taking fluorescent micrographs of the sections, those sections were fixed with 10% formaldehyde, HE staining was performed and micrographs of the same sections were taken.

### 10. Statistical analysis

Statistical significance was assessed using Tukey-Kramer multiple comparisons test. All data are expressed as the mean + standard error (SE). Values of p<0.05 were accepted as statistically significant.

## Results

### 1. Viability of the skin after pressurization

Results of quantitative evaluation of the viability of pressurized skin are shown in Fig 1. Pressurized skin samples in NSS-0, DW-0, NSS-100, DW-100 and NSS-150 showed viability, but those in DW-150, NSS-200, DW-200, NSS-1000 and DW-1000 did not.

**Fig 1:** Comparison of the viability of pressurized skin. The mean absorbance of DMEM was set as an arbitrary zero point. The absorbance levels of NSS-0, DW-0, NSS-100, DW-100 and NSS-150 were significantly higher than that of DMEM (p<0.01). The absorbance levels of DW-150, NSS-200, DW-200, NSS-1000 and DW-1000 were significantly lower than those of NSS-0, DW-0, NSS-100, DW-100 and NSS-150 (p<0.01). The absorbance level of NSS-0 was significantly higher than those of NSS-100, DW-100 and NSS-150 (p<0.01). The absorbance level of NSS-150 was significantly lower than those of NSS-100 and DW-100 (p<0.01).

After the outgrowth culture of the pressurized skin, fibroblasts were observed in NSS-0, DW-0, NSS-100, DW-100, NSS-150 and DW-150, but no cells were confirmed in NSS-200, DW-200, NSS-1000 and DW-1000 on Day 14 (Fig 2). After cultivation, the viability of pressurized skin samples in DW-150 was revitalized, but the samples pressurized at more than 200 MPa still showed no viability (Fig 3).

**Fig 2:** Micrographs of fibroblasts on Day 14. Yellow arrows indicate pressurized skin and blue arrowheads indicate fibroblasts. Scale bar: 100 μm.

**Fig 3:** Comparison of the viability of pressurized skin after cultivation on Day 14. The absorbance levels of NSS-0, DW-0, NSS-100, DW-100, NSS-150 and DW-150 were significantly higher than that of DMEM (p<0.01). The absorbance levels of NSS-200, DW-200, NSS-1000 and DW-1000 were significantly lower than those of NSS-0, DW-0, NSS-100, DW-100, NSS-150 and DW-150 (p<0.01).

### 2. Histological and immunohistochemical examination of the skin after pressurization

Epidermis of NSS-0, NSS-100 and DW-0 remained intact, but that of other groups was removed (Fig 4). No apparent damage to the extracellular matrix of the dermis was observed in all groups. Immunohistochemical staining of type IV collagen showed that the basement membranes of epidermis and capillaries in the dermis remained intact in all specimens regardless of the existence of epidermis (Fig 5). Immunohistochemical staining of vWF showed that the capillaries were intact in all groups (Fig 6).

**Fig 4:** Micrographs of HE sections of pressurized skin. Yellow arrowheads indicate the remained epidermis. Scale bar: 100 μm.

**Fig 5:** Micrographs of immunohistochemical staining of type IV collagen. Red arrowheads indicate the basement membrane of epidermis and green arrowheads indicate the basement membrane of capillaries. Scale bar: 100 μm.

**Fig 6:** Micrographs of immunohistochemical staining of vWF. Red arrowheads indicate stained capillaries. Scale bar: 100 μm.

SEM findings of pressurized skin are shown in Fig 7. The arrangement of collagen fibers was regular and they did not show apparent damage due to pressurization in all groups.

**Fig 7:** SEMs of pressurized skin. Scale bar: 100 μm.

### 3. Implantation of pressurized skin with or without CE into nude mice

HE-stained sections of implanted pressurized skin without CE on Day 14 showed that the epidermis in NSS-0, NSS-100 and DW-0 was still intact after implantation (Fig 8). The epidermis did not regenerate in the other groups in which it had been removed before implantation. CE prepared from PKH26-stained keratinocytes was implanted into those groups and took on pressurized skin in all groups except for NSS-1000 and DW-1000 (Fig 9). The infiltration of recipient cells to pressurized skin was confirmed and no apparent inflammatory response was observed (Fig 8 and Fig 9). The epidermis was not observed in NSS-1000 and DW-1000, and PKH-positive keratinocytes were scattered on the dermis and did not form epithelium in these two groups.

**Fig 8:** HE-stained sections of implanted pressurized skin without CE on Day 14. Black arrowheads indicate the epidermis of the implanted pressurized skin and red arrowheads indicate the dermis of the pressurized skin. Scale bar: 100 μm.

**Fig 9:** HE-stained sections (upper figures) and fluorescent micrographs (lower figures) of implanted pressurized skin with CE on Day 14. Yellow arrowheads show CE that took on pressurized skin on HE sections and the CE was PKH-positive in fluorescent micrographs. Scale bar: 100 μm.

## Discussion

In this study, we subjected human skin to pressurization at 100, 150, 200 and 1000 MPa for 10 minutes and showed that the skin was completely inactivated after pressurization at more than 200 MPa. When samples were placed in a bag with DW, the viability just after pressurization at 150 MPa seemed to be inactivated. However, the activity was revitalized after cultivation and the outgrowth of cells from the skin was confirmed. These findings suggest that cells present in the superficial part of the skin were inactivated by the pressure and low osmolality of DW, but cells in the deeper part were not inactivated and proliferated in the culture medium. The removal of the epidermis of DW-100 could also be explained by this. This pressure of inactivation is compatible with the findings of our previous study using cultured cells [15], and this indicates that the appropriate pressurization can inactivate all cells in skin regardless of its thickness. As for the mechanism of inactivation of cells by pressurization, it has been reported to be the result of apoptosis at around 200 MPa, and to occur through a necrotic-like pathway above 300 MPa [17,18]. It was also reported that apoptosis usually occurs after pressurization at around 100 MPa through the activation of caspase-3 via both extrinsic and intrinsic pathways [17,18]. In the clinical application of HHP, the possibility of disinfection of infectious or tumor-afflicted bone segments before their reimplantation as an autograft has been reported [19–21]. As for the inactivation of pathogens, bacteria and viruses, most of them were reported to be inactivated by HHP from 100 MPa to 300 MPa, although a much higher pressure of more than 500 MPa was needed for the inactivation of some viruses [20,21]. In addition, 1200 MPa was found to be required for the inactivation of infectious prions [22], so it would be difficult to kill all pathogens completely by using HHP. On the other hand, normal eukaryotic cells and malignant cells were reported to be more sensitive to pressure than bacteria and those cells were irreversibly impaired at a pressure of less than 350 MPa in the orthopedic field [20–23]. We showed that pressurization at 200 MPa could inactivate healthy skin, which is lower than 350 MPa. Therefore, further investigation is needed for the inactivation of skin tumor cells such as malignant melanoma or squamous cell carcinoma.

As for the damage to the extracellular matrix, our previous study using HHP at 1000 MPa did not detect any morphological damage of various tissues, such as heart valve, blood vessels and bone [11–14]. It has also been reported that the biomechanical properties of bone, tendon and cartilage remained nearly unchanged at up to 600 MPa and HHP treatment did not significantly affect extracellular matrix proteins such as fibronectin and type I collagen [20,24]. Extracellular matrix proteins such as collagen types I, II and III and proteoglycans were reported not to be modified at up to 600 MPa by immunohistochemical analysis [25]. We showed that the basement membrane of the epidermis and capillaries in the dermis remained intact at up to 1000 MPa and dermal collagen fibers showed no obvious damage or degeneration by SEM. However, CE took on dermis pressurized at up to 200 MPa, whereas it did not take on dermis pressurized at 1000 MPa. This suggests that pressurization at 1000 MPa caused some damage to the dermal matrix that was not detected histologically or immunohistologically. As for an ultra-high pressure of more than 600 MPa, there have yet to be sufficient studies about its effects on the extracellular matrix. Clarification of the damage to the pressurized dermis and the mechanism that prevents the successful take of CE are subjects for our next study.

HHP at 1000 MPa has been studied as a safe decellularization method that can inactivate tissues regardless of their thickness and hardness in a remarkably short length of time (within one hour) [10–14]. The processing time of HHP at 1000 MPa is about one hour and HHP at 200 MPa in this study requires only 20 minutes. This HHP at 200 MPa can be applied during an operation for the preparation of an inactivated autologous skin graft. In the removal of malignant skin tumors such as malignant melanoma or squamous cell carcinoma, a wide safety margin must be removed with the tumors. If we could apply HHP at 200 MPa for the intraoperative inactivation of skin tumors including the safety margin, removed skin could be reused as an autograft and we could avoid the harvesting of healthy skin from the patient’s donor site. Another clinical issue for skin reconstruction in plastic surgery is the treatment of congenital giant melanocytic nevus (GCMN). GCMN occurs in approximately one in 20,000 newborns and its most concerning complication is malignant melanoma [26,27]. In terms of the risk of melanoma, it is reported to develop in 2.8 to 8.5 percent, and 70 percent of those cases arise by the age of 13 years [26]. Therefore, surgical excision in early childhood is recommended, although it is usually difficult to excise the nevus completely because autologous skin available for skin defect after removal is limited. Dermal substitutes including AlloDerm (LifeCell Corp., Branchburg, N.J.), Integra (Integra Life Science Corp., Plainsboro, N.J.) and Pelnac (Gunze Ltd., Ayabe, Japan) in combination with a split thickness skin graft have been used for the treatment of GCMN [28,29]. However, the results achieved with skin substitutes did not provide superior form and function compared with other conventional methods [26] and the long-term efficacy of these substitutes is still controversial [3,30,31]. Skin inactivated by HHP at 200 MPa in our method can retain its native quality comparable to that of autologous dermis, and inactivated nevus in combination with autologous cultured epidermis should be a breakthrough therapy in the treatment of GCMN.

The skin inactivated after HHP at 200 MPa has cellar debris that is usually washed out in the process of preparation of decellularized tissue because this debris can cause host rejection or an immunological response [32]. The taking of cultured epidermis was not affected by such remnants in this study, even though this issue needs further investigation using nevus tissue that contains abundant nevus cells. As the next step, we plan to inactivate human nevus using HHP and investigate whether CE will take on inactivated nevus with cellular debris. In this study, we mainly explored the inactivation of human skin by pressurization at 200 MPa and compared its inactivation with pressurization at 1000 MPa, which is the pressure we have been using for decellularization. We will explore pressurization and the taking of CE using intermediate pressures, such as 400 MPa or 600 MPa, in an experiment using nevus tissue as the next step.

## Conclusion

Human skin pressurized at 200 MPa for 10 minutes was inactivated without histological damage of the dermis; this inactivated skin took after implantation into nude mice in combination with human cultured epidermis. However, CE did not take on skin pressurized at 1000 MPa, which is suggestive of damage after pressurization. Skin inactivated by our method could be a breakthrough approach in the treatment of GCMN.
